The article "The Therapeutic Effect of Coriolus versicolor Fruiting Body on STZ-Induced ICR Diabetic Mice" was published in 2022. Journal: J Healthc Eng.

# The Therapeutic Effect of *Coriolus versicolor* Fruiting Body on STZ-Induced ICR Diabetic Mice

**DOI:** 10.1155/2022/7282453

**Published:** 2022-04-15

**Authors:** Fanxin Meng, Yumiao Lin, Lifu Hu, Wei Feng, Peiwen Su, Liyan Wu

**Affiliations:** School of Pharmacy and Food Science, Zhuhai College of Science and Technology, Jinwan 519041, China

## Abstract

*Coriolus versicolor* is a natural drugs which has many pharmacological effects such as antitumor and enhanced immune activity. This paper studies the therapeutic effect of *Coriolus versicolor* fruiting body (CVFB) on streptozotocin (STZ)-induced Institute of Cancer Research (ICR) diabetic mice, the STZ solution was administered intraperitoneally at a dose of 150 mg/kg after fasting the mice, and ICR mice with fasting blood glucose >16.7 mmol/l were selected for research. Metformin was the positive control, and the dose of CVFB powder (1000 mg/kg, 2000 mg/kg, and 4000 mg/kg) for 28 consecutive days by gavage. The serum and liver of mice were collected for relevant index content testing. The results showed that CVFB can control or reduce the fasting blood glucose of mice and accelerate the rate of glucose metabolism, can reduce the levels of total cholesterol (T-CHO), triglyceride (TG), and high-density lipoprotein cholesterol (HDL-C) in mice, and regulate the abnormal symptoms of blood lipid metabolism commonly found in diabetes. It can increase the activity of superoxide dismutase (SOD) and glutathione peroxidase (GSH-Px) antioxidant enzymes and enhance the ability of antioxidative stress in diabetic mice. In the H&E staining and apoptosis experiments of pancreatic tissue, CVFB can greatly reduce the inflammatory factors present in islets, increase the islet cells, and reduce the apoptotic rate caused by diabetes. All data confirmed the therapeutic effect of CVFB on diabetic ICR mice. The present study provides a scientific basis for the development of drugs for the prevention and treatment of diabetes, it is of great significance to the in-depth study of *Coriolus versicolor.*

## 1. Introduction

According to the 9th edition of the Diabetes Map released by the International Diabetes Federation (IDF), diabetes is one of the most common chronic diseases in the world, and the number of adult patients with diabetes of the world is increasing year by year, while the number of adult patients with diabetes in China ranks first in the world, according to the noncommunicable disease.

Current research has not yet found a cure for diabetes drugs or treatment, controlling and treating diabetes are a long-term, ongoing, and slow-moving task, while most diabetes drugs have toxic side effects while treating the symptoms of hyperglycemia, long-term consumption of antidiabetic drugs will aggravate the burden on the liver and kidney, leading to a series of complications. Natural medicine is a kind of natural product with some pharmacological activities, including plants, animals, and minerals, and are easy to be absorbed and utilized by the human body and have stable effects and little toxic side effects on the body. The study found that many natural products have good hypoglycemic components, such as polysaccharides, polyphenols, flavonoids, alkaloids, and other compounds [1]. Therefore, in the prevention and treatment of diabetes, the full use of natural drug adjuvant therapy can improve the efficacy and reduce side effects.

The article "The Therapeutic Effect of Coriolus versicolor Fruiting Body on STZ-Induced ICR Diabetic Mice" was published in 2022. Journal: J Healthc Eng.

*Coriolus versicolor* is a natural drug which has many pharmacological effects such as antitumor, ant-atherosclerosis, antiaging, antioxidation, and enhanced immune activity [2–9]. At present, the research on *Coriolus versicolor* is mainly focused on macromolecular compounds such as polysaccharide, glycopeptide, and glycoprotein, but *Coriolus versicolor'*s chemical composition is very complex.

Therefore, this article studies the therapeutic effect of the CVFB on ICR diabetic mice which is caused by streptozotocin (STZ); after the treatment, glucose metabolism, lipid metabolism, and antioxidant indexes of the experimental mice were detected, as well as further pathological analysis of the pancreas. This provides a scientific basis for the development of drugs for the prevention and treatment of diabetes and is of great significance for the in-depth study of CVFB.

## 2. Materials and Methods

### 2.1. CVFB Powder and Metformin Hydrochloride Preparation

*Coriolus versicolor* fruiting body powder: origin is Heilongjiang, purchased from Johncan International, Hangzhou, China.

Metformin hydrochloride tablets: Sino-American Shanghai Squibb Pharmaceuticals Ltd.

### 2.2. Development of Diabetic Mouse Models

A total of 120 four-week-old male ICR mouses ((SPF) grade, SCXK (YUE)-2013-0002) were adaptability to fed about 2 weeks. After 18 h fast (free access to water), mice of 22 + 2 g were subjected to 150 mg/kg STZ solution intraperitoneally (except the NS group); the control group was injected with citric acid buffer; 2 h after administration, the mice were fed. After 7 days of feeding, fasting without water was done to measure fasting blood glucose. The fasting blood glucose value of mice ≥16.7 mmol/L was determined to be a successful model.

### 2.3. Drug Treatment Procedure

Diabetic mice were randomly divided into five groups with more than 12 mice in each group (to avoid death in the experiment). Normal mice served as the control group. The duration of drug administration was 28 days. Normal control group (normal saline, NS) and model group (diabetic control, DC) were given sterile normal saline gavage, and positive control group (positive control, PC) was given 200 mg/kg metformin hydrochloride by gavage; the drug group was intragastrically administrated with the CVFB at concentrations of 1000 mg/kg (low dose, LD), 2000 mg/kg (medium dose, MD), and 4000 mg/kg (high dose, HD). Routine diet was fed after administration. Water intake, food intake, weight, and fasting blood glucose were recorded regularly.

The article "The Therapeutic Effect of Coriolus versicolor Fruiting Body on STZ-Induced ICR Diabetic Mice" was published in 2022. Journal: J Healthc Eng.

### 2.4. Oral Glucose Tolerance Test (OGTT)

Oral glucose tolerance test (OGTT) is a glucose stress test used to determine whether an organism has diabetes to understand the function of pancreatic beta cells in vivo and the body's ability to regulate blood sugar. During the OGTT test, fasting without water for 6 h in the evening of the 26th day of the treatment period and fasting blood glucose values of diabetic mice in each group were measured in the morning of the 27th day. Each group was given 2 g/kg glucose by gavage at one time. Tail venous blood was taken, and blood glucose values of 30 min, 60 min, 90 min, and 120 min after glucose administration were measured by a blood glucose meter and recorded.

### 2.5. Sample Collection

At the end of the treatment period, the mice were weighed, and then mice were euthanized by ether, the blood was collected by eyeball extirpation, and the organs (liver, kidney, spleen, thymus, pancreas and heart) of the mice were collected and weighing. The pancreas was washed with cold saline and fixed with Carnoy's fluid for tissue sectioning. A small part of liver was washed with cold normal saline, and an appropriate amount of liver fragments were homogenized in cold 0.9% normal saline (liver (g):0.9% normal saline (mL) = 1 : 9). The homogenized mixture was centrifuged at 3000 RPM at 4°C for 10 min, and the supernatant was collected to obtain 10% liver homogenate. The samples were stored at −20°C.

### 2.6. Serum and Liver Homogenate Sample Index Detection

The contents of glycated serum protein (GSP), insulin (Ins), T-CHO, TG, HDL-C, low-density lipoprotein cholesterol (LDL-C), and blood urea nitrogen (BUN) in the serum and the contents of malondialdehyde (MDA), SOD, and GSH-Px in the serum and liver homogenate were detected by Nanjing Jiechen Kits (Nanjing Jiancheng Institute of Biological Engineering, Nanjing, China).

### 2.7. Pancreatic Histopathological Tests

Pancreatic tissue was fixed in Carnoy's fluid for 24 h, and the tissue was removed for dehydration, embedding, and sectioning. After the tissue sectioning was completed, some sections were stained with hematoxylin and eosin by H&E to observe the shape of pancreatic cells; the other sections were added with proteinase K and reacted with TUNEL kit (Roche) to observe the apoptosis of pancreatic cells.

The article "The Therapeutic Effect of Coriolus versicolor Fruiting Body on STZ-Induced ICR Diabetic Mice" was published in 2022. Journal: J Healthc Eng.

### 2.8. Statistical Analysis

All data are expressed as mean ± standard error (S.EM.). SPSS 20.0 software was used for statistical analysis of the data. A one-way analysis of variance (ANOVA) and multiple comparisons were combined to calculate the significance of the data. In statistics, when *p* > 0.05, it is considered no significant difference, when *p* < 0.05, it is considered significant difference, when *p* < 0.01, it is considered very significant difference, and when *p* < 0.001, it is considered extremely significant difference.

## 3. Results

### 3.1. The Effects of the CVFB on Water Intake, Food Intake, Body Weight, and Organ Index of Diabetic Mice

During the treatment period, the water and food intake in the DC group increased significantly compared with the NS group. The body weight of mice in NS group was significantly different from that in 0 days of treatment (*p* < 0.001; Table 1, No. c) and increasing rate on day 28 of the treatment period was 58.0%, while there was no significant difference in the body weight of mice in DC group.

After 28 days of treatment, the water intake in 5 groups of diabetic mice increased significantly compared with 0 days of treatment (*p* < 0.001; Table 1, No. a). The body weight of mice in the PC group and CVFB treatment group increased significantly compared with 0 days of treatment (*p* < 0.01; Table 1, No. c); compared with the DC group of mice, CVFB dosage group weight increased significantly after 28 days (29.3 ± 0.8; 29.7 ± 0.9, and 30.5 ± 1.4) having significant difference, in which the weight gain was similar to that of the positive control group (29.8 ± 0.9).

Compared with the NS group, the weight of the kidney index was significantly increased (*p* < 0.001; Table 1, No. d), the weight of the spleen, thymus, and heart index was significantly decreased (*p* < 0.001; Table 1, No. d), and the weight of the pancreas index was also decreased in the DC group.

After 28 days of administration of CVFB, it was found that CVFB could inhibit the trend of changing the direction of the organs in the DC group, and the indexes of related organs returned to normal level.

### 3.2. The Effects of the CVFB on Glucose Metabolism in Diabetic Mice

After 28 days of treatment, the fasting blood glucose concentration of diabetic mice treated with the CVFB decreased to the concentration of 0 days of treatment (*p* > 0.05; Table 2), and the fasting blood glucose concentration of the PC group was significantly different from that at 0 days of treatment (*p* < 0.05; Table 2).

The article "The Therapeutic Effect of Coriolus versicolor Fruiting Body on STZ-Induced ICR Diabetic Mice" was published in 2022. Journal: J Healthc Eng.

Mice were given 2.0 g/kg glucose solution by gavage for OGTT test. After gavage, the blood glucose of each group increased significantly. After 30 minutes, the blood glucose value of each group showed a different trend to decrease; at 60 minutes, there was a significant difference in blood glucose between the PC group and the DC group (*p* < 0.05; Figure 1), and it was observed that the PC group had a greater tendency to decrease blood sugar than the DC group; at 90 min, the blood glucose levels of the HD group and the PC group were significantly different from those of the DC group (*p* < 0.05, *p* < 0.01; Figure 1).

After 28 days of administration, the CVFB groups and the PC group all decreased the levels of GSP to a certain extent (*p* > 0.05; Figure 2(a)) and had a certain degree of decline in INS content levels and MD and HD groups and PC groups had significant differences in the decline of INS content levels (*P* < 0.05; Figure 2(b)). HOMA-IR was decreased in the HD and PC groups (*P* < 0.05; Figure 2(c)).

### 3.3. The Effects of the CVFB on Lipid Metabolism in Diabetic Mice

After treatment, the concentrations of T-CHO (*p* < 0.05; Figure 3(a)), TG, and BUN (*p* < 0.01; Figures 3(b) and 3(e)) in diabetic mice were decreased, and the content of HDL-C was significantly increased (*p* < 0.05; Figure 3(c)), indicating that CVFB groups had a certain regulatory effect on lipid metabolism in diabetic mice.

### 3.4. The Effects of the CVFB on Antioxidant in Diabetic Mice

The serum and liver homogenate of mice were tested. In the serum test, it can be seen that the SOD activities of the MD and HD groups and PC group are all increased (*p* < 0.001; Figure 4(a)). The content of MDA in the LD, MD, and HD groups and the PC group decreased (*p* < 0.05, *p* < 0.01, *p* < 0.001, *p* < 0.001; Figure 4(b)); GSH-Px activity increased in the LD, MD, and HD groups and the PC group (*P* < 0.05, *p* < 0.05, *p* < 0.01, *p* < 0.01; Figure 4(c)).

In liver homogenate, SOD activity increased in the MD and HD groups and PC group (*p* < 0.01, *p* < 0.001, *p* < 0.001; Figure 4(a)). The content of MDA was decreased in the LD, MD, and HD of the CVFB group and the PC group (*p* < 0.01, *p* < 0.001, *p* < 0.001, *p* < 0.001; Figure 4(b)). The GSH-Px activity increased in the LD, MD, and HD groups and the PC group (*p* < 0.01, *p* < 0.01, *p* < 0.001, *p* < 0.001; Figure 4(c)).

The CVFB group and the PC group had certain antioxidant effects on diabetic ICR mice, and the positive drug metformin had better antioxidant properties than the CVFB groups, but there was no significant difference between them.

The article "The Therapeutic Effect of Coriolus versicolor Fruiting Body on STZ-Induced ICR Diabetic Mice" was published in 2022. Journal: J Healthc Eng.

### 3.5. The Effects of the CVFB on Histopathology in Diabetic Mice

#### 3.5.1. H&E Staining Results of Pancreatic Tissue Sections

It can be seen from Figure 5 that the number of pancreatic islet cells in the LD group is greatly reduced, and the interior and surrounding of the pancreatic islets are infiltrated by a large number of inflammatory cells, but the borders of the pancreatic islets can still be distinguished.

The pancreatic islets of the mice in the MD group were slightly atrophy, and there were inflammatory cells around the pancreatic islets. Compared with the negative control group, the inflammatory cells were greatly reduced. The structure of pancreatic islets in the HD group is relatively complete, with obvious borders, compared with the DC group, the islet cells are significantly increased, and the inflammatory cells are greatly reduced. However, there are still more inflammatory cells on the side of the islets.

With the concentration of CVFB increased, the number of inflammatory cells gradually decreased.

#### 3.5.2. TUNEL Method to Determine the Results of Cell Apoptosis in Pancreatic Tissue

In the NS group (Figure 6), Normal cells are evenly distributed in mouse pancreatic islets; when there is inflammation, inflammatory cells are produced and pile up together; in the DC group (Figure 6), many inflammatory cell nuclei are distributed inside and outside the pancreatic islets. The *h* diagram shows that diabetes caused by STZ can cause cell apoptosis, and the apoptosis rate is significantly increased.

In the CVFB high-dose group (Figure 6), the inflammatory cells around the pancreatic islets of the mouse were significantly reduced, and the cells in the pancreatic islets were more evenly distributed. The apoptosis rate was significantly reduced (Figure 6).

## 4. Discussion

In this experiment, we used the STZ one-time high-dose injection method to build a diabetic ICR mouse model to explore the therapeutic effect of CVFB. Glucose metabolism, lipid metabolism, and antioxidant effects of diabetic ICR mice and the impact on mouse pancreas organs were analyzed by the daily living conditions.

Diabetes is a disease characterized by a relative or absolute lack of insulin, leading to hyperglycemia. Injecting large doses of STZ damages pancreatic *β*-cells, causing *β*-cell dysfunction and reducing insulin secretion, and inducing mice to become nonobese diabetic [10]. From the measurement results, we can see that CVFB can effectively control or reduce the fasting blood glucose of diabetic mice to a certain extent and reduce the levels of GSP and INS in the fasting serum. However, the sensitivity of related organs and tissues in diabetic mice to insulin is reduced, and insulin resistance promotes glucose uptake, which causes a variety of biochemical reactions in the body. Therefore, high levels of fasting plasma insulin can reflect insulin resistance [11]. The experimental results show that the HOMA-IR evaluation is reduced, indicating that CVFB can significantly improve insulin resistance and protect pancreatic *β* cells. At the same time, the OGTT test results show that CVFB can accelerate the decomposition and utilization of blood sugar and finally accelerate the glucose metabolism in diabetic mice.

The article "The Therapeutic Effect of Coriolus versicolor Fruiting Body on STZ-Induced ICR Diabetic Mice" was published in 2022. Journal: J Healthc Eng.

Diabetes is one of the most common metabolic diseases, in which abnormal lipid metabolism is often an important factor in determining the direction and status of the disease [12]. The experimental results found that CVFB can reduce the content level of T-CHO, TG, BUN, and LDL-C, increase the content level of HDL-C, accelerate the metabolism of blood lipids in diabetic mice, and regulate the disorder of lipid metabolism in the body to reduce the incidence of hyperlipidemia and also reduce the risk of coronary heart disease, atherosclerosis, and diabetes complications.

Many researchers have proved that the oxidative damage associated with diabetes is caused by the production of reactive oxygen species. Therefore, increasing the activity of antioxidant enzymes can increase the body's antioxidant defense system's response to oxidative stress [13]. The experimental results found that CVFB can effectively increase the activity of antioxidant enzymes SOD and GSH-Px in the serum and liver homogenate of diabetic mice and reduce the level of MDA. MDA is the main product of lipid peroxides, which proves that diabetes is related to oxidative stress. The pancreas is an internal organ that produces insulin and glucagon, which regulates the body's blood sugar stability. Observing the H&E staining results and the apoptosis experiment of the pancreas tissue of diabetic mice, it can be seen that compared with the NS group, the CVFB group can reduce the inflammatory factors in the pancreatic islets in the pancreas of diabetic ICR mice and improve the damaged islet structure and increase the islet cells and the apoptosis rate was significantly reduced, indicating that CVFB has a protective effect on the pancreas of diabetic ICR mice.

In this experiment, we studied the therapeutic effect of CVFB on STZ-induced ICR diabetic mice and found that diabetic mice administered with CVFB can control or reduce the blood sugar level of diabetic mice, accelerate the rate of glucose metabolism, regulate the lipid metabolism disorder and abnormal blood lipid metabolism in the body, enhance the antioxidant capacity in mice, reduce oxidative stress damage, protect the pancreas organs, and repair and adjust the function of the pancreas to regulate blood sugar balance. In this experiment, we studied the therapeutic effect of CVFB on STZ-induced ICR diabetic mice and found that diabetic mice administered with CVFB can control or reduce the blood glucose level of diabetic mice and accelerate the rate of glucose metabolism, regulate the lipid metabolism disorder and abnormal blood lipid metabolism in the body, enhance the antioxidant capacity in mice, reduce oxidative stress damage, protect the pancreas organs, and repair and regulate the function of the pancreas to regulate blood sugar balance.

The article "The Therapeutic Effect of Coriolus versicolor Fruiting Body on STZ-Induced ICR Diabetic Mice" was published in 2022. Journal: J Healthc Eng.

The above aspects show that CVFB has a therapeutic effect on diabetic mice, provides a scientific basis for the development of drugs for the prevention and treatment of diabetes, and is of great significance to the in-depth research of *Coriolus versicolor*.

## Figures and Tables

**Figure 1:** The effect of CVFB on OGTT of STZ-induced ICR diabetic mice. ###*p* < 0.001 versus NS group, ^*∗*^*p* < 0.05, and ^*∗∗*^*p* < 0.01versus DC group.

**Figure 2:** The effect of CVFB on the level of GSP (a), INS (b), and HOMA-IR (c) in the serum of STZ-induced ICR diabetic mice. ###*p* < 0.001 versus NS group. ^*∗*^*p* < 0.05 versus DC group.

**Figure 3:** The effect of CVFB on the level of T-CHO (a), TG (b), HDL-C (c), LDL-C (d), and BUN (e) in the serum of STZ-induced ICR diabetic mice. ##*p* < 0.01 and ###*p* < 0.001 versus NS group; ^*∗*^*p* < 0.05 and ^*∗∗∗*^*p* < 0.001 versus DC group.

**Figure 4:** The effect of CVFB on the level of SOD (a), MDA (b), and GSH-Px (c) in the serum and liver homogenate of STZ-induced ICR diabetic mice. ##*p* < 0.01 and ###*p* < 0.001 versus NS group; ^*∗∗*^*p* < 0.01 and^*∗∗∗*^*p* < 0.001 versus DC group.

**Figure 5:** The picture of histopathological analysis in pancreas of STZ-induced ICR diabetic mice (×400).

**Figure 6:** The picture of apoptosis analysis in pancreas of STZ-induced ICR diabetic mice (a–l).

**Table 1:** The effect of 28-day CVFB treatment on the water intake, food intake, body weights, and organ index of STZ-induced ICR diabetic mice (*n* = 11).

No.				NS	DC	LD	MD	HD	PC
	Water intake (ml)	28 days	0	7.9 ± 0.2	45.6 ± 2.2	44.2 ± 2.6	50.8 ± 1.4	44.2 ± 2.4	46.5 ± 2.3
			7	5.0 ± 0.6^*∗∗*^	46.9 ± 1.3	47.7 ± 0.8	50.0 ± 2.6	50.0 ± 4.2	50.0 ± 1.2
a			14	5.0 ± 0.6^*∗∗*^	55.6 ± 0.9^*∗∗∗*^	59.4 ± 0.8^*∗∗∗*^	64.1 ± 1.7^*∗∗∗*^	56.3.0 ± 4.6^*∗∗∗*^	56.9 ± 1.4^*∗∗∗*^
			21	6.7 ± 1.2	58.1 ± 0.7^*∗∗∗*^	57.5 ± 1.9^*∗∗∗*^	66.7 ± 2.3^*∗∗∗*^	61.3 ± 5.0^*∗∗∗*^	60.0 ± 1.5^*∗∗∗*^
			28	4.2 ± 0.3^*∗∗∗*^	62.5 ± 0.6^*∗∗∗*^	63.1 ± 1.1^*∗∗∗*^	66 ± 1.4^*∗∗∗*^	61.9 ± 3.7^*∗∗∗*^	61.8 ± 1.6^*∗∗∗*^

	Food intake (g)	28 days	0	9.4 ± 0.1	11.9 ± 0.8	10.8 ± 0.5	11.3 ± 0.2	10.7 ± 0.4	10.2 ± 0.8
			7	5.2 ± 0.2	11.0 ± 0.8	9.8 ± 0.3	9.2 ± 0.4	10.1 ± 0.6	8.1 ± 0.3^*∗*^
b			14	5.8 ± 0.2	10.2 ± 0.1	11.6 ± 0.3	11.7 ± 0.3	11.3 ± 0.5	10.2 ± 0.7
			21	5.5 ± 0.2	10.5 ± 0.2	10.4 ± 0.3	10.1 ± 0.4	9.8 ± 0.4	9.2 ± 0.9
			28	4.5 ± 0.1^*∗∗∗*^	11 ± 0.2	11.6 ± 0.2	11.0 ± 0.2	10.3 ± 0.3	9.1 ± 0.3

	Body weights (g)	28 days	0	23.1 ± 0.8	25.2 ± 1.0	24.9 ± 0.9	24.0 ± 0.8	25.9 ± 1.4	25.4 ± 1.1
			7	28.7 ± 0.6^*∗∗∗*^	23.1 ± 1.0	24.3 ± 0.7	24.2 ± 0.8	26.1 ± 1.0	24.1 ± 1.1
c			14	33.4 ± 0.6^*∗∗∗*^	26.6 ± 1.0	26.2 ± 0.9	26.9 ± 1.0^*∗*^	29.4.0 ± 1.3^*∗*^	28.6 ± 0.7^*∗*^
			21	31.6 ± 0.7^*∗∗∗*^	24.9 ± 1.0	28.25 ± 0.8^*∗∗*^	27.9 ± 0.8^*∗∗*^	25.9 ± 1.2	25.2 ± 0.4
			28 growth rate (%)	36.5 ± 0.8^*∗∗∗*^58.0	25.1 ± 1.0–0.4	29.3 ± 0.8^*∗∗*^17.7	29.7 ± 0.9^*∗∗∗*^23.8	30.5 ± 1.4^*∗∗*^17.8	29.8 ± 0.9^*∗∗*^17.3

	Organ index (mg/g)		Liver	49.4 ± 1.8	53.0 ± 1.9	50.8 ± 1.9	47.3 ± 1.6	48.9 ± 1.8^#^	49.8 ± 0.8
			Kidney	14.1 ± 0.3^###^	18.4 ± 0.4	19.9 ± 0.4^##^	18.6 ± 0.5	17.2 ± 0.4^#^	17.6 ± 0.5
d			Spleen	2.8 ± 0.3^###^	1.7 ± 0.04	1.9 ± 0.1	1.6 ± 0.1	1.5 ± 0.1	2.0 ± 0.2
			Thymus	1.0 ± 0.1^###^	0.4 ± 0.03	0.7 ± 0.1^##^	0.5 ± 0.1	0.4 ± 0.1	0.4 ± 0.04
			Pancreas	6.3 ± 0.3	5.9 ± 0.3	5.9 ± 0.4	5.6 ± 0.2	6.1 ± 0.4	6.2 ± 0.3
			Heart	4.6 ± 0.1^###^	3.6 ± 0.1	3.9 ± 0.1^#^	3.5 ± 0.1	3.8 ± 0.1	3.7 ± 0.2

^*∗*^ *p* < 0.05, ^*∗∗*^*p* < 0.01, and^*∗∗∗*^*p* < 0.001 are the comparisons between within the group and day 0; #*p* < 0.05, ##*p* < 0.01, and ###*p* < 0.001 versus DC group. Growth rate: body weights increment (day 28–day 0)/body weight (day 0)×100%.

The article "The Therapeutic Effect of Coriolus versicolor Fruiting Body on STZ-Induced ICR Diabetic Mice" was published in 2022. Journal: J Healthc Eng.

**Table 2:** The effect of 28-day CVFB treatment on the fasting blood glucose of STZ-induced ICR diabetic mice (*n* = 11).

28 days	0	7	14	21	28
NS	6.3 ± 0.2	8.5 ± 0.3^*∗∗*^	7.9 ± 0.5^*∗*^	8.4 ± 0.5^*∗∗*^	6.2 ± 0.4
DC	24.9 ± 1.3	29.1 ± 0.7^*∗*^	30.6 ± 0.8^*∗∗*^	31.6 ± 0.7^*∗∗*^	27.4 ± 0.8
LD	23.4 ± 1.2	27.8 ± 0.9^*∗*^	29.7 ± 0.8^*∗∗∗*^	28.5 ± 0.8^*∗∗*^	22.8 ± 1.1
MD	24.8 ± 0.8	30.3 ± 0.7^*∗∗*^	29.6 ± 0.7^*∗∗*^	29.7 ± 0.8^*∗*^	24.2 ± 1.7
HD	24.4 ± 1.1	26.5 ± 1.1	27.48 ± 1.1	27.9 ± 1.2	22.8 ± 1.8
PC	25.3 ± 0.9	28.9 ± 0.7^*∗*^	27.8 ± 1.0	26.7 ± 1.0	22.2 ± 1.5^*∗*^

^*∗*^ *p* < 0.05, ^*∗∗*^*p* < 0.01, and ^*∗∗∗*^*p* < 0.001 are the comparisons between within the group and day 0.

## Data Availability

The data used and analyzed during the current study are available from the corresponding author on reasonable request.
